This article has been retracted.

# Decreased miR-154 expression and its clinical significance in human colorectal cancer

**DOI:** 10.1186/s12957-015-0607-5

**Published:** 2015-06-06

**Authors:** Yang Kai, Cheng Qiang, Pan Xinxin, Zhou Miaomiao, Lin Kuailu

**Affiliations:** Department of Surgical Oncology, The First Affiliated Hospital of Wenzhou Medical College, Wenzhou, 325000 China; Department of neurology, Huai’an No. 2 Hospital, Huai’an Jiangsu Province, China

**Keywords:** MiR-154, Colorectal cancer, Prognosis, Overall survival

## Abstract

**Background:**

miRNA-154 (miR-154) has been identified as a tumor suppressor in several types of human cancers. However, its clinical significance in colorectal cancer (CRC) is still unclear. The aim of this study was to analyze the association of miR-154 expression with clinicopathologic features and prognosis in CRC patients.

**Methods:**

Quantitative RT-PCR was performed to evaluate miR-154 levels in 169 pairs of CRC specimens and adjacent noncancerous tissues. Then, the associations of miR-154 expression with clinicopathological factors or survival of patients suffering CRC were determined.

**Results:**

The expression levels of miR-154 in CRC tissues were significantly lower than those in corresponding noncancerous tissues (*P* < 0.001). Decreased miR-154 expression was significantly associated with large tumor size, positive lymph node metastasis, and advanced clinical stage. Moreover, the univariate analysis demonstrated that CRC patients with low miR-154 expression had poorer overall survival (*P* = 0.006). The multivariate analysis identified low miR-154 expression as an independent predictor of poor survival.

**Conclusions:**

These findings suggested that miR-154 downregulation may be associated with tumor progression of CRC, and that this miR may be an independent prognostic marker for CRC patients.

## Background

Colorectal cancer (CRC) ranks as the third most prevalent cancer worldwide. Despite the clinical implementation of numerous therapeutic strategies, it remains a leading cause of cancer-related deaths due to therapy resistance and metastasis [1]. Previous studies have demonstrated diverse genetic alterations in CRC, but the highly complex molecular mechanisms underlying CRC carcinogenesis and progression remain obscure. Therefore, it is necessary to search novel markers for CRC, which can accurately identify biological characteristics of tumors, improve therapeutic strategies, and predict clinical outcome.

MicroRNAs (miRs) are a class of short (about 22 nucleotides in length), endogenous, single-stranded, non-protein-coding RNAs that directly bind to the 3’-untranslated regions (3’-UTRs) of target messenger RNAs (mRNAs), leading to mRNA degradation or translational suppression [2]. Beyond the involvement in diverse biological processes, including cell growth, apoptosis, development, differentiation, and endocrine homeostasis [3], emerging evidence strongly suggests that the deregulation or dysfunction of miRs contributes to human carcinogenesis and cancer progression [4–6]. miRs can function as either oncogenes or tumor suppressors according to the roles of their target genes. In terms of CRC, abnormal expression of several miRs such as miR-27b, miR-133b, and miR-124 have been reported [7–9]. Zhang et al. found that ectopic expression of miR-224 promoted CRC tumor cell proliferation, migration, and invasion in vitro [10]. Zheng et al. indicated that downregulation of miR-132 in CRC was associated with tumor size, distant metastasis, and TNM stage [11]. Furthermore, miR-218, miR-378, miR-378a-3p, and miR-378a-5p expressions were independent prognostic factors for CRC patients [12–14]. miR-129 sensitized CRC cells to 5-FU both in vitro and in vivo [15], and miR-124 could increase the radiosensitivity of CRC cells [16]. These findings suggest that miRs act not only as diagnostic and prognostic markers but also as potential therapeutic targets of CRC.

Extensive researches have shown that miR-154 is deregulated and functions as a candidate tumor suppressor in some tumors such as hepatocellular carcinoma and prostate cancer [17, 18]. Interestingly, Xin et al. found that miR-154 was decreased in CRC tissues and cell lines [19]. Ectopic expression of miR-154 remarkably suppressed cell proliferation and colony formation, migration and invasion in CRC cells. However, the roles of miR-154 in the progression of CRC and its underlying potential to predict clinical outcome of patients with this disease remain elusive. The aim of this study was to analyze the association of miR-154 expression with clinicopathologic features and prognosis in patients suffering CRC.

## Methods

### Tissue samples and cell lines

This study was approved by the Research Ethics Committee of The First Affiliated Hospital of Wenzhou Medical College. Written informed consent was obtained from all of the patients. All specimens were handled and made anonymous according to the ethical and legal standards.

A total of 169 pairs of primary CRC and adjacent noncancerous tissues were obtained from patients who underwent surgery at The First Affiliated Hospital of Wenzhou Medical College between January 2006 and December 2008. None of the patients had received chemotherapy or radiotherapy before surgery excision. After collection, all tissue samples were immediately frozen in liquid nitrogen and stored at −80 °C until use. The patients’ information is summarized in Table 1. All of the patients received follow-up. Overall survival was defined as the time from primary surgery to death of the patient or, for living patients, the date of last follow-up.

**Table 1:** Correlation between miR-154 expression and different clinicopathological features in colorectal cancer patients

Clinicopathological features	No. of cases	miR-154 expression		*P* value
		Low (*n* = 84)	High (*n* = 85)	
Age				
<60	78	41	37	0.539
≥60	91	43	48	
Gender				
Male	98	51	47	0.534
Female	71	33	38	
Tumor size (cm)				
<5	95	39	56	0.013
≥5	74	45	29	
Histology/differentiation				
Well + moderate	88	38	50	0.091
Poor	81	46	35	
Depth of invasion				
T1 + T2	64	28	36	0.268
T3 + T4	105	56	49	
N classification				
Negative	69	24	45	0.002
Positive	100	60	40	
TNM stage				
I	30	9	21	0.004
II	39	15	24	
III	100	60	40	

### RNA extraction and quantitative real-time PCR

Total RNA was extracted from clinical specimens with Trizol reagent (Invitrogen Corp, Carlsbad, CA, USA) according to the manufacturer’s instructions. RNA concentration was measured using NanoDrop (Thermo Scientific). Ten nanograms of total RNA was transcribed into cDNAs using a TaqMan MicroRNA Reverse Transcription Kit (Applied Biosystems, Foster City, CA, USA). Real-time PCR was performed with a Taqman MicroRNA Assay Kit (Applied Biosystems) on ABI7500 real-time PCR detection system. The PCR program for detecting miRs was as follows: 50 °C for 2 min, 95 °C for 10 min, 40 cycles of 95 °C for 15 s, and 60 °C for 1 min. U6 small nuclear RNA was used as an internal control. Each sample was measured in triplicate, and the relative amount of miR-154 to U6 was calculated using the equation 2^−ΔCt^, where ΔCT = (CT_miR−154_ − CT_U6_).

### Statistics

All statistical analyses were carried out using the SPSS 16.0 software package (SPSS, Chicago, IL, USA). Data were presented as mean ± standard deviation (SD). Differences between groups were analyzed using the Student’s *t*-test or chi-square test. The postoperative survival rate was analyzed with Kaplan-Meier method, and differences in survival rates were assessed with log-rank test. A Cox proportional hazards model was used for multivariate analysis. *P* < 0.05 was considered to be statistically significant.

## Results

### Downregulation of miR-154 in human CRC tissues

The expression levels of miR-154 were detected in 169 pairs of CRC and corresponding adjacent noncancerous tissues normalized to U6 small nuclear RNA. As shown in Fig. 1, the expression levels of miR-154 in CRC tissues were found to be distinctly decreased compared to noncancerous tissues. The results showed that the relative level of miR-154 expression in CRC tissues (mean ± SD: 8.92 ± 2.12) was significantly lower than that in corresponding noncancerous tissues (mean ± SD: 19.36 ± 4.35; *P* < 0.001).

**Fig. 1:** MiR-154 expression was significantly lower in colorectal cancer samples than in the corresponding noncancerous tissues (*P* < 0.001, paired *t*-test). MiR-154 expression levels were calculated by the 2^−ΔCt^ method and normalized to U6 small nuclear RNA

### Downregulation of miR-154 associates with advanced clinicopathological features of CRC

The associations of miR-154 expression with various clinicopathological parameters of CRC tissues were analyzed. The patients were divided into two groups according to their miR-154 expression levels, using the median of miR-154 expression in all 169 patients as a cutoff: high miR-154 expression group (*n* = 85) and low miR-154 expression group (*n* = 84). As shown in Table 1, miR-154 was significantly downregulated in CRC patients with large tumor size (*P* = 0.013), positive lymph node metastasis (*P* = 0.002), and advanced clinical stage (*P* = 0.004). No significant difference was observed between miR-154 expression and patients’ age, gender, tumor differentiation, and depth of invasion.

### Downregulation of miR-154 confers poor prognosis in CRC patients

Using the Kaplan-Meier method and log-rank test, we found that the overall survival of CRC patients with low miR-154 expression was significantly shorter than those with high miR-154 expression (*P* = 0.006; Fig. 2). Besides, the survival benefits were also found in those with smaller tumor size (*P* = 0.026), early T classification (*P* = 0.032), negative N classification (*P* = 0.004), and early clinical stage (*P* = 0.015). Multivariate Cox regression analysis enrolling abovementioned significant parameters revealed that miR-154 expression (relative risk (RR) 2.825; *P* = 0.022), lymph node metastasis (RR 4.958; *P* = 0.005), and TNM stage (RR 5.232; *P* = 0.001) were independent prognostic markers for overall survival of CRC patients (Table 2).

**Fig. 2:** Kaplan-Meier survival curves of patients with colorectal cancer based on miR-154 expression status. Patients in the low expression group had significantly poorer prognosis than those in high expression group (*P* = 0.006, log-rank test)

**Table 2:** Univariate and multivariate analyses of prognostic factors in colorectal cancer

Variable	Univariate analysis			Multivariate analysis		
	HR	95 % CI	*P* value	HR	95 % CI	*P* value
Age (years)	1.632	0.761–3.534	0.215	–	–	–
Gender	1.134	0.533–2.445	0.759	–	–	–
Histological grading	1.704	0.792–3.668	0.173	–	–	–
Tumor size	2.629	1.132–5.237	0.026	2.116	0.945–4.572	0.078
Depth of invasion	2.388	1.076–5.224	0.032	1.524	0.635–3.162	0.283
Lymph node metastasis	5.395	1.986–10.655	0.004	4.958	1.923–10.115	0.005
Clinical staging	2.973	1.202–6.488	0.015	5.232	1.998–12.685	0.001
MiR-154	3.178	1.436–9.356	0.006	2.825	1.006–5.132	0.022

## Discussion

Dysregulation of miRs has been demonstrated to be involved in tumorigenesis and progression in various types of tumor; however, elucidation of their potential roles in CRC remains in the early stage of development. In the current study, we found that miR-154 was downregulated in human CRC tissues compared with noncancerous tissues. We also found that decreased miR-154 expression in CRC tissues was significantly correlated with aggressive clinicopathological features. Moreover, Kaplan-Meier analysis showed that CRC patients with low miR-154 expression tend to have shorter overall survival. The multivariate analysis confirmed low miR-154 expression as a significant risk factor for overall survival, indicating that miR-154 might be involved in CRC progression and could be used as a potential prognostic biomarker. To the authors’ knowledge, this is the first study to investigate the clinical significance of miR-154 in a large number of CRC patients.

miR-154 is located on human chromosome 14q32, which is frequently lost in human cancers [20–22], and miR-154 downregulation has been reported to play important roles in cancer progression. For instance, Wang et al. found that restoration of intracellular miR-154 suppressed tumor cell malignance and the G1/S transition in hepatocellular cancer cells [18]. Zhu et al. indicated low miR-154 expression levels in primary prostate cancer compared with nonmalignant samples [23]. Forced expression of miR-154 significantly reduced the migratory and invasive capabilities of prostate cancer cells. Our study confirmed miR-154 downregulation in CRC tissues, which is consistent with the previous study of Xin et al. [19]. The current data also demonstrated that miR-154 might be related to the clinical outcome of patients with CRC, while Xin’s article reported the tumor-suppressive function of miR-154 in CRC at the cell level. Taken together, these results revealed that loss of miR-154 might play a critical role in cancer formation and progression, and miR-154 could act as a novel target for cancer diagnosis and therapy.

It is now clear that miRs execute their oncogenic or tumor suppressor functions by regulating the expression of target genes [24]. Xin et al. identified the toll-like receptor 2 (TLR2) as a direct target of miR-154 in CRC cells [19]. In their study, inhibition of TLR2 performed similar effects with miR-154 overexpression on the biological behavior of CRC cells, and overexpression of TLR2 could significantly reverse the tumor-suppressive effects of miR-154 on CRC cells. However, there is no “one-to-one” connection between miRs and target mRNAs. An average miR can have more than 100 targets [25]. Conversely, several miRs can converge on a single transcript target [26]. TLR2 is not the only miR-154 target dysregulated in CRC. Other functional targets of miR-154, such as cyclin D2 (CCND2), also modulate CRC pathogenesis [27, 28]. Therefore, the potential regulatory circuitry afforded by miR-154 is enormous, and the accurate mechanisms on how miR-154 influences CRC progression need further clarification.

## Conclusions

In summary, our present study showed that miR-154 was downregulated in CRC tissues, and low miR-154 expression was significantly correlated with aggressive clinicopathological features and worse prognosis. However, the molecular mechanisms underlying miR-154 and the regulation of CRC carcinogenesis have not been fully elucidated. Therefore, this study is hypothesis generating, and further prospective analysis is worth doing.
